RETRACTED

# Effect of Roxadustat on Factors Associated with Renal Fibrosis and Efficacy

**DOI:** 10.1155/2022/4764254

**Published:** 2022-08-08

**Authors:** Fangfang Zheng, Peng Zhang, Mingzuo Zhao, Jinna Wang, Xiaohong Xu, Chi Zhang, Li Zhang

**Affiliations:** ^1^Department of Pharmacy, The Affiliated Suqian Hospital of Xuzhou Medical University, Suqian Hospital of Nanjing Drum Tower Hospital Group, Suqian, Jiangsu 223800, China; ^2^Department of General Surgury, The Affiliated Suqian Hospital of Xuzhou Medical University, Suqian Hospital of Nanjing Drum Tower Hospital Group, Suqian, Jiangsu 223800, China; ^3^Department of Nephrology, The Affiliated Suqian Hospital of Xuzhou Medical University, Suqian Hospital of Nanjing Drum Tower Hospital Group, Suqian, Jiangsu 223800, China; ^4^Department of Nursing, The Affiliated Suqian Hospital of Xuzhou Medical University, Suqian Hospital of Nanjing Drum Tower Hospital Group, Suqian, Jiangsu 223800, China

## Abstract

**Objective:**

We investigated the effect of roxadustat on factors associated with renal fibrosis and efficacy*. Methods*. Sixty patients meeting the inclusion criteria between January 2021 and October 2021 were equally distributed into observation (roxadustat) group and control (Erythropoietin) group. Then, the expression of serum hypoxia-inducible factor 1-alpha (HIF-1*α*), transforming growth factor-*β* (TGF-*β*1), vascular endothelial growth factor (VEGF), fibronectin (FN), and collagen Ⅳ (C-IV) was compared at different time points (baseline, 2-week follow-up, and 4-week follow-up). The improvement degree of hemoglobin (Hb) and the change level of iron parameters and hepcidin were also compared between the two groups*. Results*. In the roxadustat group, the expression of HIF-1*α* at 2 weeks was significantly higher than the baseline and approached the baseline value at 4 weeks. At 4 weeks, TGF-*β*1 and FN expression was significantly lower than baseline. In addition, the improvement of Hb in the roxadustat group was significantly higher than that in the control group at 4 weeks, and the change of ferritin, transferrin, and hepcidin indexes from baseline was better than in the control group.

**Conclusion:**

After giving roxadustat, it can change the expression of HIF-1*α*, TGF-*β*1, and FN. Its efficacy is superior to EPO, which is worthy of clinical application.

## 1. Introduction

Renal anemia is a common complication of chronic kidney disease (CKD). It often occurs in patients with CKD after stage 3, when renal function has significantly decreased [1]. Renal anemia is associated with some adverse outcomes, including reduced quality of life for patients, increased incidence of cardiovascular disease, increased hospital admissions, cognitive impairment, and death [2, 3]. The kidney is the main source of erythropoietin (EPO), produced by interstitial fibroblasts around peritubular capillaries and proximal tubules. EPO stimulates the production of red blood cells in the bone marrow and drives hemoglobin homeostasis, and EPO concentrations are 10-100 times lower in patients with renal anemia compared to those with similar anemia. In addition, erythropoiesis inhibitors, shortened red blood cell survival time, and iron deficiency due to uremia can also lead to nephrogenic anemia [4]. The current drugs commonly used to treat renal anemia are erythropoietin and iron, but there is a risk of causing hypertension, oxidative stress and cardiovascular disease, and allergic reactions [5].

RETRACTED

Roxadustat (FG-4592, FibroGen) is a hypoxia-inducible factor (HIF) prolyl hydroxylase inhibitor that stabilizes HIF-1*α* subunits, causing increased HIF transcriptional activity, which leads to functional activation of early-response target genes encoding proteins such as EPO and EPO receptor, enzymes such as heme synthetase and proteins that promote iron absorption and transport, resulting in coordinated erythropoiesis [6]. In recent years, roxadustat has been studied more frequently for the treatment of CKD combined with anemia [7], but studies on renal fibrosis have not been reported so far. Renal fibrosis is the most common pathological manifestation of CKD [8]. Different levels of HIF-1*α* in the body have different effects on renal fibrosis [9]. Previous studies have shown that in the early stage of CKD, HIF-1*α* helps prevent damage from ischemia and hypoxia damage, which can also delay the progression of renal fibrosis by regulating the expression of downstream target genes [10]. However, when the HIF-1*α* expression significantly increases and exceeds a certain value, it possibly aggravates renal fibrosis and promotes the development of end-stage renal disease [11]. Therefore, this study was conducted to observe whether a small increase in HIF-1*α* induced further renal fibrosis after the administration of roxadustat.

Renal fibrosis is caused by increased synthesis and decreased degradation of extracellular matrix due to multiple factors, and the pathogenesis includes various cytokines, vasoactive substances, and inflammatory cells [12]. Among them, transforming growth factor-*β* (TGF-*β*1) is the most critical factor contributing to the formation and development of renal fibrosis [13]. Extracellular matrix components are very complex, and fibronectin (FN) and collagen IV (C-IV) are the main components, which can better reflect the interstitial fibrosis of the kidney and are often used as a clinical test for chronic kidney disease [14]. Vascular endothelial growth factor (VEGF) is necessary to participate in glomerular and tubular hypertrophy and endothelial cell proliferation in the kidney, and downregulation of VEGF leads to the development of glomerulosclerosis and tubulointerstitial fibrosis [15]. Therefore, the degree of renal fibrosis can be reflected by detecting of the levels of these factors in the serum.

RETRACTED

Based on the above studies, clarifying whether increased HIF-1*α* expression after roxadustat administration inducing further renal fibrosis is a question that needs to be addressed. Before this, it is necessary to observe the change of factors associated with renal fibrosis in the serum of patients.

## 2. Methods

### 2.1. Patients

A total of 60 patients enrolled between January 2021 and October 2021 in this study met the following conditions. (1) The patients were diagnosed with renal anemia with CKD and were not currently undergoing dialysis, which met the diagnostic criteria for the 2017 version of the “Guidelines for screening, diagnosis and prevention of chronic kidney disease” and “Chinese expert consensus on diagnosis and treatment of renal anemia.” The diagnostic of renal anemia was as follows: The patients have CKD. And the hemoglobin is at the following levels: adults living in sea-level areas, male hemoglobin (Hb) <130 g/L, nonpregnant women Hb<120 g/L, and pregnant women <110 g/L; and the diagnostic criteria for CKD were: epidermal growth factor receptor (eGFR) < 60 ml (min/1.73 m^2^); albuminuria ≥ 30 mg/24 h; abnormal urinary sediment; structural and histological abnormalities observed on imaging, and a history of kidney transplantation for more than 3 months. Second, the patients were aged ≥18 years. Thirdly, the patients received no EPO treatment in the last 4 weeks. The exclusion criteria were as follows: an inability to actively cooperate with medical staff for treatment and combined chronic diseases of the heart, brain, or other parts of the body; malignant tumors; or incomplete medical records.

The target number of patients was reference to the previous data and literature [12] and patients with chronic kidney disease who had been previously diagnosed as renal anemia and had not received dialysis were measured. Consider that there may be patients who do not want to be enrolled or lost to follow-up and other circumstances. Based on this, the sample size of this study was determined to be 60. In this study, SPSS 25.0 software was used to generate random numbers, and participants were randomly divided into roxadustat group or EPO group.

### 2.2. Study Design

Thirty patients were randomly assigned to the roxadustat group who received roxadustat for renal anemia. Thirty patients in the control group received EPO for renal anemia. Patients completed at least 4 weeks of medication follow-up surveys. This is based on a small sample of patients who had been treated with roxadustat for renal anemia which showed a significant increase in efficacy from baseline at approximately 2 weeks, while patients with chronic kidney disease had different complications with changes in renal function. In order to reduce the influencing factors, follow-up periods were set at 2 weeks and 4 weeks.

RETRACTED

Dosing method: The dosage is according to the instructions. Eligible patients received roxadustat (FG-4592, FibroGen Medical Technology Development Company, Ltd., 50 mg and 20 mg). The starting dose of roxadustat was either 100 mg (in patients weighing 45 to <60 kg) or 120 mg (in patients weighing ≥60 kg), three times per week for 4 weeks. The control group was given EPO for injection (Shanghai Kaimao Pharmaceutical & Biological Co., Ltd., 4000 IU/bottle) at an initial dose of 100-150 IU/(kg-body weight) per week, and the dose was adjusted according to the trend of hemoglobin level and changes. The hemoglobin level was maintained in the range of 90.0–120.0 g/L. The use of oral iron therapy was allowed; intravenous iron therapy was prohibited except as a rescue therapy. Rescue therapy included intravenous iron, blood transfusion, or erythro-poiesis-stimulating agents (or a combination of these treatments) in patients with a hemoglobin level less than 80.0 g per liter.

Patients who received roxadustat treatment lasted for 4 weeks, and blood was collected for enzyme-linked immunosorbent assay (ELISA) examination.

ELISA sample processing: Three milliliters of blood were collected into an anticoagulant tube at the endpoints of baseline, 2 weeks, and 4 weeks. The supernatant was collected using a pipette. The supernatant that could not be collected was first centrifuged, and then, the supernatant was collected. The supernatant samples were centrifuged (centrifuge model XK80-A) at 3000 rpm for 10 min. The ELISA kit (Nanjing Sempega Biotechnology Co., Ltd.) was used to examine the indicators related to renal fibrosis, measured according to the manufacturer's protocol.

### 2.3. Evaluation Criteria and Data Collection

The patients in this study come from the department of nephrology in our hospital. The doctor and I identified enrolled patients, and the nurse was responsible for blood drawing. The basic characteristics of patients were recorded: age, sex, drug dosage at the start of the target duration, adjustment of drug dosage and remedial measures during treatment, and iron use. Data on biochemical indexes were also collected, including blood fat, kidney function, hemameba, albumin, blood, and glucose. In addition, some of the indicators observed are as follows: changes in the following indexes were observed at baseline, 2 weeks, and 4 weeks of drug administration. (1) HIF-1*α*, TGF-*β*1, FN, C-IV, and VEGF, measured by ELISA; (2) Efficacy indicator: Hb; (3) Iron metabolism-associated indicators: serum ferritin, TRF transferrin (TRF), and hepcidin (iron-regulating factor); (4) Adverse drug reactions (ADR): related indexes of kidney detected before and after treatment and the occurrence of ADR in patients during drug administration.

RETRACTED

### 2.4. Statistical Analysis

SPSS 25.0 statistical software was used to analyze the data. The normal distribution of measurement data was expressed as mean ± standard deviation (SD). Nonnormally distributed data are represented by median and quartile. The *T*-test or Wilcoxon test was used to compare the measurement data between the two groups. The number and percentage of various cases were used to describe the counting index, and the *χ*2 test or Fisher's exact test was used to compare the data. Changes before and after treatment were compared with baseline values by paired analysis of *T*-test or Wilcoxon test. The significance level was set at *P* < 0.05.

## 3. Results

### 3.1. Patient Characteristics

A total of 60 patients who met the inclusion criteria were collected between January 2021 and October 2021, including 30 patients in the roxadustat group who received roxadustat for renal anemia. 30 patients in the control group received EPO for renal anemia. Patients completed at least 4 weeks of medication follow-up surveys. All patients successfully completed the study (Figure 1). The background information of the patients is shown in Table 1. After analysis by the statistical software SPSS, the basic data of the 2 groups of patients were not significantly different.

### 3.2. The Expression Levels of Serum HIF-1*α* at Different Time Points

To observe the serum HIF-1*α* levels in patients during roxadustat treatment for renal anemia, we measured the serum HIF-1*α* levels in patients using ELISA (Figure 2). Initially, there was no significant difference in the roxadustat group compared with baseline values (*P* > 0.05). In the second week, HIF-1*α* serum levels reached 0.95 ± 0.21 *μ*mol/L in the roxadustat group, significantly higher than the baseline value of 0.47 ± 0.21 *μ*mol/L in the control group (*P* < 0.05); at weeks four, HIF-1*α* serum levels decreased to baseline levels in the roxadustat group (*P* > 0.05).

### 3.3. The Expression of Renal Fibrosis-Related Indicators

The expression of VEGF and C-IV was not significantly different from baseline values at both 2 and 4 weeks of treatment in both the roxadustat group and the control group (*P* > 0.05). Compared with baseline, TGF-*β*1 and FN levels did not change significantly after 2 weeks of treatment, but at week 4, both TGF-*β*1 and FN levels were significantly lower (*P* < 0.05) (Figure 3).

RETRACTED

### 3.4. Hemoglobin Levels

At four weeks, one patient's hemoglobin exceeded the target value in roxadustat group, and no patient's hemoglobin exceeded the target value in the EPO group. During the treatment period, the mean change from baseline in the hemoglobin level was an increase of 19.4 ± 8.3 g/L in the roxadustat group and an increase of 14.3 ± 10.6 g/L in the EPO group (*P* < 0.05) (Figure 4).

### 3.5. Iron Metabolism and Hepcidin

At four weeks, the change from baseline in the ferritin decreased significantly (*P* < 0.05), and the decrease was significantly higher in the roxadustat group than in the control group (*P* < 0.05). In the roxadustat group, transferrin increased significantly (*P* < 0.05) from baseline after 4 weeks of treatment and the change was significantly higher than in the control group (*P* <0.05), while transferrin did not change significantly in the control group (*P* > 0.05). For the hepcidin, there was a significant decrease from baseline after 4 weeks of treatment (*P* < 0.05) and a significantly higher change than in the control group (*P* < 0.05), while there was no significant change in hepcidin in the control group before and after treatment (*P* > 0.05) (Table 2).

### 3.6. Safety

There were no significant changes in serum creatinine (Scr) and blood urea nitrogen (BUN) before and after administration (*P* > 0.05) (Table 3). No serious adverse reactions were found in the two groups. One case of nausea and hypertension was reported in each group, and one case of weakness was reported in the roxadustat group. There was no significant incidence of adverse reactions between the two groups (*P* > 0.05) (Table 4).

## 4. Discussion

Previous studies have shown that HIF-1*α* has both beneficial and detrimental effects in chronic kidney disease [16, 17]. The pharmacological action of roxadustat is to increase HIF-1*α* expression by mimicking hypoxia in vivo and inhibiting prolyl hydroxylase [18]. This study aimed to observe the influence of roxadustat on factors associated with renal fibrosis in the blood of patients.

Serum fibrosis indicators reflect the progression of the fibrotic disease [19–21]. The main pathological feature of chronic renal fibrosis is the accumulation of proteins such as extracellular matrix (ECM), FN, and C-IV [22]. VEGF is a downstream target gene of HIF-1*α*, and the effect of VEGF is related to the isoform and the amount of secretion. A moderate amount of VEGF secretion can promote the formation of new blood vessels, improve local tissue blood supply, and reduce renal nephrogenic fibrosis [23]. In this study, the results showed that HIF-1*α* levels increased significantly at 2 weeks and decreased at 4 weeks, converging to baseline values after treatment with roxadustat. This indicates that HIF did not increase continuously after roxadustat administration. In addition, at two and four weeks, VEGF and C-IV collagen did not change significantly from baseline, while FN decreased significantly from baseline at 4 weeks. This suggests that roxadustat may have a protective effect on the kidney.

RETRACTED

There is considerable evidence that TGF-*β*1 is heavily upregulated in clinical and animal models of kidney injury and that hypoxia in the body increases TGF-*β*1 production, directly stimulating renal fibrosis [24]. Our results showed that TGF-*β*1 expression was significantly lower at 4 weeks of treatment compared to baseline, possibly due to a decrease in TGF-*β*1 expression induced by HIF-1*α*. There is another possibility since it is affected by better control of renal anemia by roxadustat. Of course, the purpose of this project is to understand whether roxadustat has an effect on the expression of some factors. The specific mechanism of influence needs further study.

This study was to observe the changes of Hb in the two groups to reflect the therapeutic effect of renal anemia. The results showed that although HIF-1*α* was significantly higher at 2 weeks and then tended to the baseline level, Hb levels were consistently higher, and the changes in Hb in the roxadustat group at 4 weeks were significantly higher than those in the control group. And then, we analyzed Hb's important influencing factors iron metabolism indexes and hepcidin. The result showed that hepcidin levels decreased significantly, and transferrin increased compared to baseline values after 4 weeks of roxadustat administration. This is likely due to the direct effect of roxadustat on the stabilization of HIF levels. TRF is a well-studied HIF target with two HIF binding sites in its 5′ enhancer region [25, 26]. On the other hand, similar changes may be due to a decrease in hepcidin, which in turn promotes intestinal absorption of iron and improves macrophage iron release to form TRF [27]. A decrease in ferritin levels was also observed after 4 weeks of treatment compared to baseline values, probably due to an increase in the effective iron utilization and thus a decrease in stored iron manifested as a decrease in ferritin levels. It is suggested that the regulatory advantage of roxadustat on iron metabolism indicators and Hepcidin is closely related to have a better efficacy compared to the control group.

RETRACTED

However, this study also has the shortcoming that only the results of 2 reviews after dosing were observed. Further research is needed to determine the long-term effects and mechanisms after roxadustat administration.

## 5. Conclusions

In conclusion, HIF-1*α* expression was significantly increased after roxadustat treatment and then to normal. Roxadustat significantly reduced FN and TGF-*β*1 levels in the serum of patients with CKD combined with anemia, which in turn improved renal fibrosis. Therefore, compared with EPO, roxadustat is not only convenient to take orally and has good efficacy, but also may have a protective effect on renal fibrosis. It is worthy of clinical use.

## Figures and Tables

**Figure 1:** Patients characteristics.

**Figure 2:** The expression level of serum HIF-1*α* in patients. Note: ^∗^*P* < 0.01 vs. baseline.

**Figure 3:** Changes in expression of TGF-*β*1, FN, C-IV, and VEGF. Note: ^∗^*P* < 0.05 vs. baseline.

**Figure 4:** Hemoglobin levels. Comparison with baseline values, ^∗^*P* < 0.05.

**Table 1:** Patient baseline characteristics.

Characteristic	Roxadustat (*n* = 30)	Control (*n* = 30)	*P* value
Age (years)	55.3 ± 10.5	54.4 ± 8.3	0.590
Male sex, *n* (%)	14 (46.7%)	16(53.3%)	0.606
Weight (kg)	63.3 ± 10.8	65.1 ± 9.9	0.431
Diabetics, *n* (%)	8 (26.7%)	9 (30%)	0.774
Hypertensives, *n* (%)	21 (70%)	23 (76.7%)	0.559
Iron users, *n* (%)	19 (63.3%)	24 (56.7%)	0.152
TC (mmol/L)	4.4 ± 1.4	4.2 ± 1.3	0.498
Albumin (g/L)	38.0 ± 4.3	38.7 ± 4.9	0.468
TG (mmol/L)	1.6 ± 0.8	1.7 ± 0.7	0.664
LDL-C (mmol/L)	2.4 ± 0.8	2.5 ± 0.7	0.472
HDL-C (mmol/L)	1.1 ± 0.5	1.2 ± 0.4	0.178
Leukocytes (×10^9^/L)	7.2 ± 2.6	6.8 ± 1.9	0.481
Fasting glucose (mmol/L)	6.1 ± 1.3	5.8 ± 0.8	0.336
eGFR (ml/L)	32.8 ± 13.4	33.8 ± 11.4	0.755
BUN(mmol/L)	18.70 ± 8.60	17.80 ± 9.37	0.351

**Table 2:** Changes in iron metabolism and hepcidin levels in the two groups of patients.

	Roxadustat points	Roxadustat (*n* = 30)	Control (*n* = 30)
Serum ferritin (ng/mL)	Baseline	273.81 ± 119.39	260.0 ± 84.2
	Wk 4	170.28 ± 93.19^∗^	224.0 ± 82.2^∗^
	Change	−103.53 ± 75.25^#^	−36.0 ± 79.9

Transferri (g/L)	Baseline	1.80 ± 0.36	1.79 ± 0.56
	Wk 4	2.27 ± 0.46^∗^	1.94 ± 0.45
	Change	0.47 ± 0.46^#^	0.15 ± 0.58

Hepcidin (ng/mL)	Baseline	93.9 ± 53.0	84.9 ± 38.3
	Wk 4	51.6 ± 37.7^∗^	68.3 ± 37.3
	Change	42.3 ± 43.1^#^	16.6 ± 45.2

^∗^ *P* < 0.05 vs baseline; #*P* < 0.05 vs Wk 4.

**Table 3:** Changes of renal function indexes before and after treatment.

	Roxadustat points	Roxadustat (*n* = 30)	Control (*n* = 30)
Scr (*μ*mol/L)	Baseline	348.67 ± 167.92	331.20 ± 152.46
	Wk 4	341.87 ± 160.37	336.88 ± 158.86

BUN (mmol/L)	Baseline	18.70 ± 8.60	17.80 ± 9.37
	Wk 4	18.62 ± 9.85	18.13 ± 7.41

RETRACTED

**Table 4:** The occurrence of adverse reactions in the two groups.

	Roxadustat	Control	*P* value
Nausea	1 (4.35)	1 (5.00)	0.92
Weakness	1 (4.35)	0	0.345
Hypertension	1 (4.35)	1 (5.00)	0.92

## Data Availability

The data used to support the findings of this study are available from the corresponding author upon request.
